# Improved Cardiac Function and Attenuated Inflammatory Response by Additional Administration of Tirofiban during PCI for ST-Segment Elevation Myocardial Infarction Patients

This article has been retracted.

**DOI:** 10.1155/2021/8371996

**Published:** 2021-06-16

**Authors:** Jing Zhang, Guomin Ding

**Affiliations:** Department of Cardiology, People's Hospital of Anji, Huzhou, China

## Abstract

ST-segment elevation myocardial infarction (STEMI) is one of the acute coronary syndromes, and it is the main cause of cardiac death worldwide. The purpose of this study was to investigate whether tirofiban improves cardiac function and attenuates inflammatory response in STEMI patients undergoing percutaneous coronary intervention (PCI). From May 2016 to May 2019, a total of 124 patients who admitted into our hospital due to STEMI fulfilled inclusion and exclusion criteria and were randomly assigned to PCI + tirofiban and PCI groups, 62 cases per groups. Intravenous administration of 10 *μ*g kg^−1^ min^−1^ tirofiban was performed 30 min prior to PCI. During PCI, tirofiban infusion through a micropump with 0.15 *μ*g kg^−1^ min^−1^ lasted for 48 h. It was found that the PCI + tirofiban group was significantly different from the PCI group in total corrected TIMI frame count (CTFC) after PCI (15.88 ± 5.11 vs. 22.47 ± 6.26, *P* < 0.001). At day 7 and day 30 post-PCI, a significant time-dependent decrease in the levels of brain natriuretic peptide (BNP), cardiac troponin I (cTnI), and creatine kinase isoenzyme (CK-MB) in both groups was observed after PCI (*P* < 0.001). More importantly, the patients in the PCI + tirofiban group had much lower levels of BNP, cTnI, and CK-MB compared with those in the PCI group at days 7 and 30 post-PCI (*P* < 0.001). At day 7 following PCI, the left ventricular ejection fraction (LVEF) was statistically higher in the PCI + tirofiban group than in the PCI group (*P* < 0.05). At day 30 post-PCI, increased LVEF concomitant with reduced left ventricular end diastolic diameter (LVEDD) and left ventricular end systolic diameter (LVESD) was observed in the PCI + tirofiban group compared with the PCI group. At day 7 and day 30 post-PCI, both groups displayed a time-dependent decline in the levels of C reactive protein (CRP), tumor necrosis factor-*α* (TNF-*α*), interleukin-6 (IL-6), and procalcitonin (PCT) after PCI (*P* < 0.05). Additionally, the patients in the PCI + tirofiban group had lower levels of CRP, TNF-*α*, IL-6, and PCT compared with those in the PCI group at days 7 and 30 post-PCI (*P* < 0.05). All patients in the PCI + tirofiban and PCI groups were followed up for 12 months by outpatient or telephone after discharge. There were fewer patients with LVEF < 50% in the PCI + tirofiban group than the PCI group (*P*=0.044). Furthermore, it was found that the incidence rate of major adverse cardiovascular events (MACEs) in the PCI + tirofiban group was evidently lower than that in the PCI group (12.90% vs. 29.03%, *P*=0.028). Taken together, our data suggest that additional administration of tirofiban could improve cardiac function and attenuate inflammatory response in STEMI patients undergoing PCI, which is worthy of promotion in clinic.

## 1. Introduction

Acute coronary syndromes (ACS), as the general term of ischemic myocardial disease, are due to the coronary atherosclerotic plaque rupture and vascular occlusion causing secondary thrombosis, and the degree of myocardial injury is associated with the area of myocardium covered by the vessel and the duration of occlusion [1, 2]. The ACS involves non-ST-segment elevation myocardial infarction, ST-segment elevation myocardial infarction (STEMI), and myocardial infarction [3]. Among them, STEMI covered about 36% of ACS cases according to the Global Registry of Acute Coronary Events. Similar findings have been found in a developing country, which indicates that STEMI accounts for 37% of ACS cases in the Jakarta Acute Coronary Syndrome registry database [4, 5]. STEMI is the leading cause of premature death worldwide, and with great morbidity and mortality [6]. At present, the reperfusion therapy and preventive measures are associated with reducing the mortality of STEMI [7]. According to the recently published European Society of Cardiology guidelines 2017, the management and modification of STEMI compared with those in 2012 reveals that the percutaneous coronary intervention (PCI) remains a significant contributor to effective therapy in patients with STEMI [8]. It can be performed soon after diagnosis, and with lower mortality, reinfarction, and stroke rates compared with thrombolysis therapy [9, 10]. But during the PCI perioperative period, some complications, such as the coronary artery perforation, accidental vascular closure, stent deformation, and wire fracture, occurred occasionally due to the incision site and intubation of the coronary artery [11], and for the ACS patients, it might cause acute myocardial infarction and bleeding complications [12]. Nowadays, the dual antiplatelet therapy with aspirin and clopidogrel after PCI was widely used as a well-established efficacy treatment, which prevented the major ischemic events. However, the appropriate dosage and administration timing of the clopidogrel still remain controversial before PCI [12]. Usually, the acute MI might lead to heart failure, which can be indicated by brain natriuretic peptide (BNP). BNP is a hormone produced by the heart and a marker of heart failure. The increasing concentration of BNP is positively related to the degree of heart failure [13]. The other factors involving creatine kinase isoenzyme (CK-MB), myoglobin (MYO), cardiac troponin I (cTnI), and cardiac troponin T (cTnT) are associated with acute MI, and the higher these concentrations, the severer the disease [14]. The STEMI presents the secondary thrombosis, and the platelet is a crucial part in thrombosis by forming platelet aggregation [15]. Glycoprotein IIb/IIIa receptor inhibitors (GPIs), blocking the binding of fibrinogen to receptors through selectively blocking the GP receptors on the surface of platelets, are considered to be the most effective inhibitors of platelet activity [15, 16]. The 2009 STEMI guidelines of the European Society of Cardiology recommended that GPIs were considered the second treatment after the standard dual antiplatelet therapy [17]. The ischemic events and thrombotic complications have been reduced when GPIs were given to STEMI patients underwent PCI [18, 19]. The tirofiban as one kind of reversible GPIs is commonly used in the cardiovascular surgery, with a result of reducing infarct size and the incidence of major adverse cardiovascular events [20]. The purpose of this study was to investigate whether tirofiban improves cardiac function and attenuates inflammatory response, preventing STEMI patients from heart injury.

## 2. Materials and Methods

### 2.1. Study Population and Patient Selection

Patients who fulfilled the diagnosis of STEMI in accordance with the 2017 European Society of Cardiology (ESC) Guidelines for the management of acute myocardial infarction in patients presenting with ST-segment elevation [21] were eligible for enrollment. Other inclusion criteria were tolerance to PCI, onset time to PCI < 12 h, and grade 0–1 according to thrombolysis in myocardial infarction (TIMI) tests. The main exclusion criteria were age > 75 years; more than class III according to the New York Heart Association (NYHA) classification [22]; pregnancy or lactation period; severe coagulation dysfunction, severe anemia, and thrombocytopenia; recent experience of cerebral hemorrhage or subarachnoid hemorrhage or a history of ischemic stroke within a week; suspected aortic dissection or aneurysm; severe liver and kidney dysfunction; and engagement in other trials. The study was approved by the Ethics Committee of our hospital, and all patients provided written informed consent.

### 2.2. Diagnosis of STEMI

In accordance with the 2017 ESC Guidelines for the management of acute myocardial infarction, the patients diagnosed with STEMI should meet the following conditions: (a) oral nitroglycerin affords no relief on the chest pain that lasts for more than 30 min and symptoms such as dyspnea, sweating, and nausea occur; (b) the onset time less than 12 h; (c) ST-segment elevation more than 0.1 mV in two or more contiguous leads revealed on the electrocardiogram; and (d) 2-time elevations of sensitive and specific biomarkers, such as cTnI and CK-MB, than the normal.

### 2.3. Study Design

Patients orally took aspirin (300 mg/d; H20120236; specification: 100 mg; Bayer Healthcare Co., Ltd., Germany) and clopidogrel (300 mg/d; H20000542; specification: 25 mg; Shenzhen Salubris Pharmaceuticals Co., Ltd., China) and received intravenous bolus of unfractionated heparin (UFH) with 0.1 mg kg^−1^ d^−1^ dosage prior to PCI. Intravenous administration of 10 *μ*g kg^−1^ min^−1^ tirofiban (H20090328; specification: 50 mL: 12.5 mg; Lunan Better Pharmaceutical Co., Ltd., Linyi, Shandong, China) was performed 30 min prior to PCI. During PCI, tirofiban infusion through a micropump with 0.15 *μ*g kg^−1^ min^−1^ lasted for 48 h. After PCI, patients were given subcutaneous injection of 1 mg/kg low-molecular-weight heparin (H20010300; specification: 1 mL: 5000 IU; Hainan Unipul Pharmaceutical Co., Ltd., China) twice a day on consecutive 7 days followed by administrations of aspirin (100 mg/d) and clopidogrel (75 mg/d) for at least 18 months and optional drugs such as statins and angiotensin-converting enzyme inhibitors as patients required.

### 2.4. Endpoints

The venous blood (5 mL) was collected from each patient and placed into EDTA-contained tubes at admission, 7 days, and 30 days post-PCI. After centrifugation, the plasma and serum was extracted, respectively. The plasma level of BNP was detected by the full-automatic immunoluminescent analyzer using a commercial available kit (Maxim Biotechnology, Fuzhou, Fujian, China). The concentration of cTnI was examined by immunoassay (Elecsys 1020; Boehringer Mannheim Diagnostics, Germany), and the activity of CK-MB was examined by the immune inhibition method (Synchron CX9; Beckman Coulter, USA). The serum levels of C reactive protein (CRP), tumor necrosis factor-*α* (TNF-*α*), interleukin-6 (IL-6), and procalcitonin (PCT) were detected using commercial available kits (Nanjing Bidi Biotechnology, Jiangsu, China). The left ventricular ejection fraction (LVEF), left ventricular end diastolic diameter (LVEDD), and left ventricular end systolic diameter (LVESD) of all patients were examined by Color Doppler Ultrasound with frequency set as 1–3 MHz (Vivid7 Dimension; General Electric Company, USA). Immediate efficacy of PCI was assessed by TIMI tests, corrected TIMI frame count (CTFC), TIMI myocardial perfusion grade (TMPG), and ST-segment elevation changes. All-cause death and major adverse cardiovascular events (MACEs) such as cardiac death; nonfatal MI; angina pectoris recurrence with revascularization, acute stent thrombosis, subacute thrombosis, and target vessel restenosis; and stroke were recorded.

### 2.5. TIMI, CTFC, and TMPG

TIMI flow is classified into 3 grades. TIMI 0 grade represents a total occlusion of blood vessels without antegrade flow; TIMI 1 grade refers to a weak antegrade flow with incomplete filling of the distal coronary bed; TIMI 2 grade, also partial reperfusion, indicates a slow antegrade blood flow with complete distal filling; and TIMI 3 grade, also full reperfusion, reveals a normal antegrade flow with complete filling of the distal coronary bed. The count from the first frame to the last frame is defined as TIMI frame count. The first frame shows the stable process from the first contact of contrast media on the inner wall of the coronary artery to the staining of vessel diameter more than 70%. The last frame reveals the contrast media reaches the distal anatomical landmark. The coronary artery involves left anterior descending artery (LAD), left circumflex artery (LCX), and right coronary artery (RCA). In general, the LAD is slightly longer than the LCX and the RCA. But it is necessary to divide the frame count of LAD by 1.7 so as to get the corrected TIMI frame count (CTFC). The CTFC detection should be performed when the patients were kept in the position where the coronary artery is completely exposed. The frame count of LCX and LAD was performed in the right anterior oblique and caudal projection. The RCA count was conducted in the left anterior oblique and cephalic projection. In order to ensure the frame count is correct, the counting was performed by two professional doctors independently and taken the average value. TMPG contains 4 levels: TMPG0 indicating no contrast in the myocardium; TMPG1 indicating slow entrance of contrast agents into the myocardium followed by contrast in the myocardium or sustained contrast in the infarct related artery (IRA) after next sequence; TMPG2 indicating delays in entrance of contrast agents into the myocardium and clearance, an increased myocardial density in the IRA, and presence of contrast agents in 3 cardiac cycles; and TMPG3 indicating normal contrast in the myocardium and clearance of contrast agents within 2 to 3 cardiac cycles.

### 2.6. Follow-Up

The patients were followed up for 12 months by outpatient or telephone after discharge. All-cause death and major adverse cardiovascular events (MACEs) such as cardiac death; nonfatal MI; angina pectoris recurrence with revascularization, acute stent thrombosis, subacute thrombosis, and target vessel restenosis; and stroke were recorded. All patients were observed by coronary computed tomography or coronary angiography.

### 2.7. Statistical Analysis

All data were processed using SPSS 20.0 software (IBM Corporation, Somers, New York, USA). Measurement data were described as mean ± standard deviation (s.d.) and analyzed by *t*-tests. Counting data were described as percentage and analyzed by chi-square tests. A level of *P* < 0.05 was considered statistically significant.

## 3. Result

From May 2016 to May 2019, a total of 124 patients who admitted into our hospital due to STEMI fulfilled predefined inclusion and exclusion criteria and were randomly assigned to PCI + tirofiban and PCI groups, 62 cases per groups. The PCI + tirofiban group contained 51 males and 11 females, and they were aged from 55 to 72 years with an average age of 64.18 ± 3.84 years. The PCI group included 49 males and 13 females, and they were aged from 54 to 74 years with an average age of (65.19 ± 4.14) years. According to the NYHA classification, the PCI + tirofiban group had 20 cases of class I, 29 cases of class II, and 13 cases of class III; and the PCI group had 23 cases of class I, 31 cases of class II, and 8 cases of class III. Other baseline variables of included STEMI patients by group are listed and compared in Table 1. There was no significant difference concerning gender, age, NYHA classification, body mass index (BMI), smoking history, hypertension, diabetes mellitus, onset time, systolic blood pressure (SBP), diastolic blood pressure (DBP), and heart rate (HR) between the two groups (*P* > 0.05).

All patients were given coronary angiography and PCI. The time of door to balloon was 85.54 ± 21.46 min in the PCI + tirofiban group and 82.73 ± 25.85 min in the PCI group, without significant difference (*P*=0.511). The numbers of patients with single-vessel disease, two-vessel disease, and three-vessel disease were 24, 18, and 20, respectively, in the PCI + tirofiban group and were 30, 16, and 16 in the PCI group, showing no significant difference (*P*=0.541). In the PCI + tirofiban group, the infarcted artery was LAD in 29 cases, LCX in 11 cases, and RCA in 22 cases; and in the PCI group, the infarcted artery was LAD in 28 cases, LCX in 9 cases, and RCA in 25 cases. No significant difference existed regarding the distribution of infarcted arteries between the two groups (*P*=0.815). The length and diameter of stent were 23.12 ± 6.95 mm and 2.96 ± 0.41 mm, respectively, in the PCI + tirofiban group and were 22.95 ± 4.82 mm and 2.91 ± 0.38 mm, respectively, in the PCI group. Still no significant difference existed between the two groups (*P*=0.875; *P*=0.483). Among 124 STEMI patients, 122 patients (98.39%) were successfully stented. Two patients failed to receive stents but received thrombus aspiration or balloon dilatation.

Myocardial perfusion and ST-segment elevation changes were compared to reflect immediate efficacy of PCI between the PCI + tirofiban and PCI groups prior to and post-PCI. The two groups exhibited no significant difference on TIMI grade prior to PCI (*P* > 0.05). There were 56 cases of TIMI grade 3 in the PCI + tirofiban group and 59 cases in the PCI group after PCI, showing no significant difference between two groups (*P* > 0.05). The PCI + tirofiban group had 3 cases of no-reflow, and the PCI group had 7 cases after PCI, without significant difference (*P* > 0.05). Considering the total CTFC after PCI, it was found that the PCI + tirofiban group was significantly different from the PCI group (15.88 ± 5.11 vs. 22.47 ± 6.26, *P* < 0.001, Table 2). According to stratification by culprit vessel, the CTFCs of LAD, LCX, and RCA were all remarkably lower in the PCI + tirofiban group than in the PCI group after PCI (*P* < 0.05). As listed in Table 2, 42 cases with TMPG3 were found in the PCI + tirofiban group and 31 cases with TMPG3 was found in the PCI group following PCI (*P*=0.047). As for ST-segment depression > 50%, no notable difference existed between the PCI + tirofiban and PCI groups (*P* > 0.05).

When assessed with cardiac function, the levels of BNP, cTnI, and CK-MB were examined in STEMI patients undergoing PCI in the presence or absence of intravenous administration of tirofiban. Increased levels of BNP, cTnI, and CK-MB are indicative of impaired cardiac function. The two groups exhibited no significant difference in the levels of BNP, cTnI, and CK-MB before PCI (BNP: 212.54 ± 139.77 vs. 210.23 ± 140.83; cTnI: 2.45 ± 0.58 vs. 2.61 ± 0.55; CK-MB: 88.23 ± 24.25 vs. 87.44 ± 23.52; *P* > 0.05). At day 7 and day 30 post-PCI, a significant time-dependent decrease in the levels of BNP, cTnI, and CK-MB in both groups was observed after PCI; the lower levels of BNP, cTnI, and CK-MB were implied in both groups at day 30 post-PCI than at day 7 post-PCI (*P* < 0.001). More importantly, as listed in Table 3, the patients in the PCI + tirofiban group had much lower levels of BNP, cTnI, and CK-MB than those in the PCI group at days 7 and 30 post-PCI (*P* < 0.001). Furthermore, we recorded the LVEF, LVEDD, and LVESD of STEMI patients undergoing PCI in the presence or absence of intravenous administration of tirofiban. No significant difference was found in the LVEF, LVEDD, and LVESD of STEMI patients between the two groups prior to PCI (*P* > 0.05). At day 7 following PCI, there was still no statistical difference on the values of LVEDD and LVESD between the two groups (*P* > 0.05), whereas the LVEF was statistically higher in the PCI + tirofiban group than in the PCI group (*P* < 0.05). Compared with day 7 following PCI, the higher LVEF was recorded in both groups at day 30 post-PCI. As for LVEDD and LVESD, the PCI + tirofiban group had reduced LVEDD and the PCI group had increased LVESD at day 30 post-PCI compared with day 7 post-PCI (*P* < 0.05). However, there was no significant difference in terms of LVESD in the PCI + tirofiban group and LVEDD in the PCI group between day 7 and 30 post-PCI (*P* > 0.05). At day 30 post-PCI, increased LVEF concomitant with reduced LVEDD and LVESD were observed in the PCI + tirofiban group compared with the PCI group (*P* < 0.05, Table 4).

With regard to inflammatory response, the levels of CRP, TNF-*α*, IL-6, and PCT were examined and determined in STEMI patients undergoing PCI in the presence or absence of intravenous administration of tirofiban. The two groups exhibited no significant difference concerning the levels of CRP, TNF-*α*, IL-6, and PCT before PCI (*P* > 0.05). At day 7 and day 30 post-PCI, both groups displayed a time-dependent decline in the levels of CRP, TNF-*α*, IL-6, and PCT after PCI (*P* < 0.05). Additionally, the patients in the PCI + tirofiban group had lower levels of CRP, TNF-*α*, IL-6, and PCT compared with the PCI group at day 7 and 30 post-PCI (*P* < 0.005, Figure 1).

All patients in the PCI + tirofiban and PCI groups were followed up for 12 months by outpatient or telephone after discharge. There were fewer patients with LVEF < 50% in the PCI + tirofiban group than the PCI group (*P*=0.044). Furthermore, it was found that the incidence rate of MACEs in the PCI + tirofiban group was evidently lower than that in the PCI group (12.90% vs. 29.03%, *P*=0.028, Table 5).

## 4. Discussion

STEMI represents one of the essential clinical manifestations of ACS [23]. PCI, as early reperfusion therapy, has been the leading treatment for STEMI for over years and continued to develop [24]. However, the STEMI patients underwent PCI do not always end up with the best outcome [25, 26]. Therefore, adjuvant anticoagulant and antiplatelet drugs are necessary to maintain epicardial and microvascular circulation [27]. They are commonly used to promote intracoronary thrombolysis and related to the decreasing microvascular occlusion and the relapse rate of ischemia [22, 28, 29]. Tirofiban, as one type of GPIs, has been considered one of the effective antiplatelet drugs acting in the veins and coronary artery and have significantly contributed to the therapy in STEMI for decades [30, 31].

This study aimed at finding out the effects of intravenous tirofiban on the cardiac function and inflammatory response for STEMI patients during PCI. There has been more evidence indicating that tirofiban was relevant with declined infarct size and reduced rate of thrombotic incidents [32]. A variety of factors including BNP, cTnI, cTnT, and CK-MB are associated with the cardiac function. The BNP concentration is a contributor to the diagnosis of heart failure [33]. The use of tirofiban in STEMI patients with TIMI 2 or TIMI 3 flow revealed a lower increase in BNP and CRP values, which deduced that the tirofiban had the function of inhibiting the rise of BNP and CPR [34]. The cardiac troponin complex comprises three subunits of troponin I, T, and C. It makes a number of significant contributions to the muscle work, and the testing of cardiac troponin has been the standard diagnosis of ACS and non-ACS myocardial injury [35, 36]. In addition, the cTnI is the central target of signal complexes targeting myofilaments, which plays an important role in regulating cardiac function [37]. The was some evidence that revealed that the increased concentration of cTnT was related to the all-cause mortality, and the elevated concentration of cTnI was relevant with the cardiovascular mortality for the non-ACS patients [38]. As a biomarker of myocardial injury, CK-MB has potential auxiliary detection value in clinic [39]. A research found out that the highest levels of CK-MB and lactic dehydrogenase were indicated in the deaths caused by ischemic heart disease [40]. In this analysis, we found, at day 7 and 30 after PCI, a decreasing trend on the BNP concentration in the PCI + tirofiban group and the PCI group, and the BNP was found to be declined more in the PCI + tirofiban group than the PCI group. The concentrations of cTnI and CK-MB were much lower in the PCI + tirofiban group than those in the PCI group. The findings showed the additional administration of tirofiban might be able to relieve the heart injury for STEMI patients. The left ventricular systolic function and diastolic function are related to the LVEF, LVEDD, and LVESD [41]. The study demonstrated that at day 30 after PCI, the LVEF, LVEDD, and LVESD values in the medium-dose group treated with 10  *μ*g/kg tirofiban were superior to those in the control group treated without tirofiban, and the LVEF in the medium-dose group was higher than that in the low-dose group treated with 5 *μ*g/kg tirofiban [42]. We found that there was no significant difference on the LVEDD and LVESD in the PCI + tirofiban group and the PCI group at day 7 after PCI, but the LVEF value was higher in the PCI + tirofiban group compared with the PCI group. At day 30 after PCI, these values in both groups were superior to that at day 7 after PCI, and the patients in the PCI + tirofiban group were with higher LVEF, lower LVEDD, and LVESD compared with those in the PCI group. Tirofiban has been commonly used in the treatment of STEMI, but the standard of clinical dosage has not been widely accepted. Recently, a study has indicated that the incidence and mortality of hemorrhage in AMI patients were positively correlated with the dose of antiplatelet drugs [43].

The STEMI might be a contributor to the immune system disorder, and the inflammatory factors such as CRP, TNF-*α*, IL-6, and PCT are associated with the immune system. Some studies have shown that TNF-*α* and IL-6 levels were higher for the children with viral infection compared with those with bacterial infection, which might deduce that the severe disease was related to the higher expression of TNF-*α* and IL-6 [44]. The CRP is a protein of acute systemic inflammation, which acts as a major marker of inflammation [45], and the elevated baseline CRP levels help measure infection and tissue damage and monitor the progression of chronic diseases [46]. The PCT is a biomarker of inflammation, which is generally increased in the bacterial infection [47]. In this study, our data showed, at day 7 and day 30 post-PCI, both groups displayed a time-dependent decline in the levels of CRP, TNF-*α*, IL-6, and PCT after PCI. Additionally, the patients in the PCI + tirofiban group had lower levels of CRP, TNF-*α*, IL-6, and PCT than those in the PCI group at days 7 and 30 post-PCI. The outcomes revealed that the intravenous tirofiban relieved inflammatory response and enhanced immunity. Hence, the choice of appropriate dose is still controversial. The initial dosage at 10 *μ*g kg^−1^ min^−1^ and continuous injection at 0.15 *μ*g kg^−1^ min^−1^ were administered in this study, but more research should be done on the incidence and mortality of hemorrhage.

In conclusion, tirofiban administration significantly reduced the BNP, cTnI, and CK-MB levels, which were more obvious at day 30 after PCI, and attenuated the inflammatory reaction in STEMI patients undergoing PCI. The LVEF was improved more for STEMI patients undergoing PCI with tirofiban administration. It may reveal that the additional administration of tirofiban was superior to the administration of aspirin and clopidogrel for STEMI patients undergoing PCI. Hence, tirofiban is worthy of further clinical promotion in the treatment of STEMI.

## Figures and Tables

**Figure 1:** Comparison of the levels of CRP, TNF-*α*, IL-6, and PCT between the PCI + tirofiban and PCI groups before PCI, at days 7 and 30 following PCI. A total of 124 patients with STEMI were randomly assigned to PCI + tirofiban and PCI groups, 62 cases per groups. ^*∗*^, ^#^*P* < 0.05 compared with before PCI and day 7 after PCI. CRP, C reactive protein; TNF-*α*, tumor necrosis factor-*α*; IL-6, interleukin-6; PCT, procalcitonin.

**Table 1:** Baseline variables of the included STEMI patients by group.

	PCI + tirofiban group	PCI group	*P*
Gender (male, *n* (%))	51 (82.26%)	49 (79.03%)	0.649
Age (years)	64.18 ± 3.84	65.19 ± 4.14	0.161
NYHA classification			0.480
Class I (%)	20 (32.26%)	23 (37.10%)	
Class II (%)	29 (46.77%)	31 (50.00%)	
Class III (%)	13 (20.97%)	8 (12.90%)	
BMI (kg/m^2^)	24.74 ± 4.10	24.53 ± 4.21	0.779
Smoking history (%)	43 (69.35%)	45 (72.58%)	0.692
Hypertension (%)	52 (83.87%)	49 (79.03%)	0.488
Diabetes mellitus (%)	23 (37.10%)	20 (32.26%)	0.571
Onset time (h)	5.38 ± 1.69	5.51 ± 1.88	0.686
SBP (mmHg)	142.02 ± 26.12	140.49 ± 23.45	0.933
DBP (mmHg)	83.89 ± 15.73	82.59 ± 16.71	0.656
HR (time/min)	85.46 ± 20.43	87.29 ± 19.44	0.610

A total of 124 patients with STEMI were randomly assigned to PCI + tirofiban and PCI groups, 62 cases per groups. NYHA, New York Heart Association; BMI, body mass index; SBP, systolic blood pressure; DBP, diastolic blood pressure; HR, heart rate.

**Table 2:** Myocardial perfusion and ST-segment elevation changes were compared to reflect immediate efficacy of PCI between the PCI + tirofiban and PCI groups prior to and post-PCI.

	PCI + tirofiban group	PCI group	*P*
TIMI grade (*n* (%))	56 (90.32%)	59 (95.16%)	0.300
No-reflow (*n* (%))	3 (4.84%)	7 (11.29%)	0.187
Total CTFC (mean ± s.d.)	15.88 ± 5.11	22.47 ± 6.26	<0.001
CTFC of LAD (mean ± s.d.)	17.12 ± 5.75	22.14 ± 6.25	<0.001
CTFC of LCX (mean ± s.d.)	13.97 ± 2.10	21.01 ± 4.89	<0.001
CTFC of RCA (mean ± s.d.)	15.76 ± 2.19	20.54 ± 4.22	<0.001
TMPG3 (*n* (%))	42 (67.74%)	31 (50.00%)	0.047
ST-segment depression > 50%	50 (80.65%)	44 (70.97%)	0.208

A total of 124 patients with STEMI were randomly assigned to PCI + tirofiban and PCI groups, 62 cases per groups. TIMI, thrombolysis in myocardial infarction; CTFC, corrected TIMI frame count; LAD, left anterior descending artery; LCX, left circumflex artery; RCA, right coronary artery; TMPG, TIMI myocardial perfusion grade.

**Table 3:** The levels of BNP, cTnI, and CK-MB in STEMI patients in the PCI + tirofiban and PCI groups at day 7 and 30 following PCI.

Group	BNP (ng/mL)		cTnI (ng/mL)		CK-MB (IU/L)	
	Day 7 after PCI	Day 30 after PCI	Day 7 after PCI	Day 30 after PCI	Day 7 after PCI	Day 30 after PCI
PCI + tirofiban group	100.36 ± 10.32^*∗*^	80.21 ± 8.65^*∗*^^#^	1.05 ± 0.09^*∗*^	0.66 ± 0.05^*∗*^^#^	29.88 ± 4.89^*∗*^	18.22 ± 1.28^*∗*^^#^
PCI group	114.12 ± 12.12^*∗*^	92.24 ± 12.35^*∗*^^#^	1.87 ± 0.17^*∗*^	1.12 ± 0.12^*∗*^^#^	35.73 ± 5.04^*∗*^	27.39 ± 4.11^*∗*^^#^
*P*	<0.001	<0.001	<0.001	<0.001	<0.001	<0.001

A total of 124 patients with STEMI were randomly assigned to PCI + tirofiban and PCI groups, 62 cases per groups. ^*∗*^, ^#^*P* < 0.05 compared with before PCI and day 7 after PCI. BNP, brain natriuretic peptide; cTnI, cardiac troponin I; CK-MB, creatine kinase isoenzyme.

**Table 4:** Cardiac function comparison between the PCI + tirofiban and PCI groups at days 7 and 30 following PCI.

Group	LVEF (%)		LVEDD (mm)		LVESD (mm)	
	Day 7 after PCI	Day 30 after PCI	Day 7 after PCI	Day 30 after PCI	Day 7 after PCI	Day 30 after PCI
PCI + tirofiban group	55.36 ± 8.21	60.21 ± 6.21^*∗*^	48.36 ± 4.12	44.12 ± 3.24^*∗*^	36.24 ± 4.34	36.87 ± 4.65
PCI group	46.21 ± 6.21	50.21 ± 4.23^*∗*^	50.02 ± 4.24	48.24 ± 3.04	37.21 ± 4.65	43.21 ± 3.54^*∗*^
*P*	<0.001	<0.001	0.655	0.029	0.232	<0.001

A total of 124 patients with STEMI were randomly assigned to PCI + tirofiban and PCI groups, 62 cases per groups. ^*∗*^*P* < 0.05 compared with before PCI. LVEF, left ventricular ejection fraction; LVEDD, left ventricular end diastolic diameter; LVESD, left ventricular end systolic diameter.

**Table 5:** The incidence rates of MACEs between the PCI + tirofiban and PCI groups 12 months following PCI.

	PCI + tirofiban group	PCI group	*P*
LVEF < 50%	11 (17.74%)	19 (30.65%)	0.040
MACEs	9 (14.52%)	19 (30.65%)	0.032
Recurrent angina pectoris	7	13	
Recurrent MI	1	3	
Malignant arrhythmia	1	1	
Heart failure	0	1	
Cardiac death	0	1	

A total of 124 patients with STEMI were randomly assigned to PCI + tirofiban and PCI groups, 62 cases per groups. LVEF, left ventricular ejection fraction; MACE, major adverse cardiovascular event.

## Data Availability

The data used to support the findings of this study are included within the article.
